The article "Correlation between Serum LP-PLA2 and sST2 Levels and the Condition of Patients with Acute Heart Failure and Their Prognostic Value" was retracted in 2023. Reasons: unreliable results or conclusions; concerns about the data; concerns about the peer review; concerns about the citations.

# Correlation between Serum LP-PLA2 and sST2 Levels and the Condition of Patients with Acute Heart Failure and Their Prognostic Value

**DOI:** 10.1155/2021/8267776

**Published:** 2021-10-18

**Authors:** Junguo Zhu, Zhongbao Ruan, Li Zhu

**Affiliations:** Department of Cardiology, Taizhou People's Hospital, Taizhou, Jiangsu 225300, China

## Abstract

Acute heart failure (AHF) occurs mostly in the elderly, which is a syndrome that occurs in the later stages of the development of cardiovascular disease. Due to the sharp decline in the patient's heart function, the patient has a high mortality rate and a poor prognosis, which seriously threaten the life safety of the elderly. Therefore, early diagnosis of AHF and timely treatment are extremely important. Lipoprotein-associated phospholipase A2 (LP-PLA2) is a newly discovered cardiovascular-specific inflammatory marker, which is closely related to the formation and progression of atherosclerotic plaque and the occurrence and development of coronary heart disease. Soluble growth stimulation expression gene 2 (sST2) protein is a protein produced under the induction of mechanical stress in cardiomyocytes. It can act as a decoy receptor to mediate the interleukin-33 (IL-33)/ST2 signaling pathway to bind to IL-33, thereby reducing the myocardial protective effect and leading to myocardial remodeling. The purpose of this study was to explore the serum LP-PLA2 and sST2 levels in AHF patients and to analyze their correlation with the disease and their prognostic value. The results showed that the levels of serum LP-PLA2 and sST2 were increased in AHF patients, and the levels of serum LP-PLA2 and sST2 in patients with adverse prognostic events were higher than those in patients without adverse prognostic events. The levels of serum LP-PLA2 and sST2 are closely related to the degree of patients' illness, among which the combined prediction of AHF patients with LP-PLA2 and sST2 has the highest value, which is worthy of promotion.

## 1. Introduction

Acute heart failure (AHF) refers to the acute onset or aggravated left heart dysfunction that leads to reduced myocardial contractility and increased heart load, resulting in increased pulmonary circulation pressure, leading to syndromes such as pulmonary circulatory congestion and cardiogenic shock [1, 2]. AHF is a syndrome in the later stage of cardiovascular disease. Clinically, AHF is mainly manifested as dyspnea, fatigue, loss of appetite, and other symptoms, accompanied by lung rale, jugular irritation, edema, and other signs. AHF mostly occurs in the elderly. Due to the sharp decline in the heart function of patients, the fatality rate is high and the prognosis is poor, which seriously threaten the life safety of the elderly [3, 4]. Therefore, early diagnosis of AHF and timely treatment are extremely important. Lipoprotein-associated phospholipase A2 (LP-PLA2) is a newly discovered cardiovascular-specific inflammatory marker, which is closely related to the formation and progression of atherosclerotic plaque and the occurrence and development of coronary heart disease [5, 6]. LP-PLA2 mainly exists in the form of binding with lipoprotein particles, forming oxidized free fatty acids and lysophospholipid choline through hydrolysis of oxidized phospholipids, activating the expression of various inflammatory factors, participating in the body's inflammatory response, and promoting the formation and progression of plaque. It plays a decisive role in the formation and progression of atherosclerosis and ultimately leads to plaque rupture and cardiovascular events [7, 8]. LP-PLA2 is an independent predictor of cardiovascular events. It can hydrolyze platelet-activating factor and lose its activity, reduce the body's inflammatory response, and have anti-inflammatory and antiatherosclerotic effects. However, most clinical studies have shown that it mainly participates in the inflammatory response of the body and plays a role in promoting the inflammatory response of the body, promoting the occurrence and development of atherosclerosis, and leading to the secondary cardiovascular events of rupture [9, 10]. At present, studies on LP-PLA2 and cardiovascular disease mainly focus on plaque progression, acute coronary syndrome, and prognosis, and there is no correlation study between LP-PLA2 and heart failure. Previous studies have shown that growth-stimulating expression gene 2 (ST2) protein is a myocardial protective gene, which can be rapidly expressed at high levels when myocardial cells are subjected to certain stimuli, such as pressure/volume load, ischemia, hypoxia, and reperfusion. Thus, it plays a cardioprotective effect such as antagonizing cardiomyocyte hypertrophy and apoptosis, inhibiting myocardial fibrosis, and improving myocardial tissue function. Some scholars define it as a mechanical stress-induced cardiomyocyte functional protein [11, 12]. sST2 can act as a decoy receptor to mediate the binding of the interleukin-33 (IL-33)/ST2 signaling pathway to IL-33, thereby reducing myocardial protection and leading to myocardial remodeling [13, 14]. This article aims to explore the serum LP-PLA2 and sST2 levels in AHF patients and analyze their correlation with the disease and their prognostic value. The specific report is as follows.

## 2. Materials and Methods

### 2.1. Patients

A total of 154 AHF patients admitted to our hospital from March 2016 to December 2019 were selected as the observation group. The inclusion criteria were as follows: all meet the diagnostic criteria of AHF [15]; age ≥60 years; accompanied by sudden dyspnea, pulmonary rales, peripheral edema, etc.; in line with the New York Heart Association (NYHA) cardiac function classification standards [16], cardiac functions II to IV; clinical data are complete. The exclusion criteria were as follows: those with congenital heart disease; those with acute coronary syndrome; those with cardiac, hepatic, and renal insufficiency; those with autoimmune or systemic infectious diseases; those with end-stage malignant tumors; those with primary thyroid disease; those with shedding during follow-up. There were 98 NYHA grade II patients, 38 NYHA grade III patients, and 18 NYHA grade IV patients. According to NYHA cardiac function grading criteria, the observation group was divided into two subgroups: the mild group (grade II) with 98 cases and the severe group (grades III and IV) with 56 cases. In the severe group, 4 cases died due to critical condition during hospitalization, and the remaining were 52 cases. In the same period, 126 healthy subjects were selected as the control group. There was no statistical difference between the two groups in general information (*P* > 0.05), and they were comparable, as shown in Table 1.

### 2.2. Serum LP-PLA2 and sST2 Level Detection

In both groups, 4 ml of fasting venous blood was collected within 24 hours of admission for testing. Enzyme-linked immunosorbent assay was used to detect serum LP-PLA2 and sST2 levels. Relevant test kits were purchased from Shanghai Enzyme-Linked Biotechnology Co., Ltd., and operations were carried out in strict accordance with the instructions.

### 2.3. Follow-Up and Event Definition

After discharge from the hospital, all patients in the observation group were followed up for 1 year, and the patient's readmission or death due to heart failure was set as the adverse prognostic event. According to whether they have adverse prognostic events, they were divided into two subgroups: event group (*n* = 44) and no event group (*n* = 106).

### 2.4. Statistical Method

The results of this experiment were statistically analyzed by SPSS 20.0 (SPSS Co., Ltd., Chicago, USA). Count data were expressed by rate, and chi-square test was used for their comparison between groups. Measurement data were expressed by mean ± standard deviation, and *t*-test was used for their comparison between groups. Spearman's correlation analysis was used for correlation analysis. The ROC curve was used to analyze the predictive value of serum LP-PLA2 and sST2 levels on the prognosis of AHF patients. *P* < 0.05 indicates that the difference is statistically significant.

## 3. Results

### 3.1. Comparison of Serum LP-PLA2 and sST2 Levels between the Two Groups

The levels of serum LP-PLA2 and sST2 in the observation group ((179.62 ± 35.39) ng/ml and (105.45 ± 21.69) pg/ml) were higher than those in the control group ((80.43 ± 16.58) ng/ml and (48.26 ± 10.08) pg/ml) (*P* < 0.05), as shown in Figure 1.

### 3.2. Comparison of Serum LP-PLA2 and sST2 Levels in Patients with Different Cardiac Function Grades

The levels of serum LP-PLA2 and sST2 in the severe group ((235.18 ± 19.05) ng/ml and (132.09 ± 26.42) pg/ml) were higher than those in the mild group ((150.14 ± 20.71) ng/ml and (91.02 ± 15.36) pg/ml) (*P* < 0.05), as shown in Figure 2.

### 3.3. Comparison of Serum LP-PLA2 and sST2 Levels in Patients with Different Prognoses

The levels of serum LP-PLA2 and sST2 in the event group ((247.56 ± 30.48) ng/ml and (142.54 ± 28.12) pg/ml) were higher than those in the no event group ((156.09 ± 21.63) ng/ml and (94.31 ± 13.05) pg/ml) (*P* < 0.05), as shown in Figure 3.

### 3.4. Correlation between Serum LP-PLA2 and sST2 Levels and Patient's Condition

Spearman's correlation analysis showed that serum LP-PLA2 and sST2 levels were directly positively correlated with NYHA cardiac function classification (*r* = 0.804, *r* = 0.781, *P* < 0.001); that is, both were positively correlated with the patient's condition, as shown in Table 2.

### 3.5. The Predictive Value of Serum LP-PLA2 and sST2 Levels on the Prognosis of Patients

ROC curve results show that the AUC of serum LP-PLA2 predicting the prognosis of AHF patients was 0.760 (95% CI: 0.680–0.840). When the best cutoff value was 165.42 ng/ml and Youden index was 0.402, the sensitivity was 95.30%, and the specificity was 44.90%. The AUC of serum sST2 predicting the prognosis of AHF patients was 0.734 (95% CI: 0.649–0.818). When the best cutoff value was 82.62 pg/ml and Youden index was 0.379, the sensitivity was 76.70%, and the specificity was 61.20%. The combination of the two predicts the prognosis of AHF patients with the AUC of 0.811 (95% CI: 0.738–0.884). When the Youden index was 0.513, the sensitivity was 86.00%, and the specificity was 65.30%, as shown in Table 3 and Figure 4.

## 4. Discussion

AHF is one of the common critical illnesses in the cardiovascular department, and it is the final outcome of a variety of cardiovascular diseases. AHF is most common with left heart failure. Acute pulmonary congestion causes breathing difficulties. In severe cases, cardiogenic shock or even death may occur, with a higher mortality rate [17–19]. The pathogenesis of AHF originates from the heart itself or factors other than the heart. The main pathophysiological mechanisms include the following: (1) malignant pathophysiological cycle: decompensation occurs when the myocardium cannot maintain sufficient circulating blood volume due to acute attacks such as acute severe myocardial injury, acute myocardial infarction, afterload-variable time/variable force/relaxation imbalance, and chronic heart failure. (2) Myocardial stunning: it refers to the hypofunction of the heart caused by persistent myocardial ischemia, but the cardiac insufficiency still exists in a short time after the improvement of myocardial ischemia. (3) Myocardial hibernation: it refers to the hypofunction of the heart caused by severe coronary ischemia, but the morphology and function of myocardial cells are still normal [20–22]. Researchers have found that brain natriuretic peptide (BNP), NT-pro BNP, and other important diagnostic biochemical markers of heart failure are restricted by age, sex, liver and kidney dysfunction, and other factors, resulting in the interference of the test results. Moreover, the exclusion value of BNP and other indicators is higher than the diagnostic value which is also an important reason for many years of challenges. The above conditions make their clinical value limited. Therefore, it is extremely important to find new biochemical markers to diagnose and predict the prognosis of patients.

LP-PLA2 is a newly discovered cardiovascular-specific inflammatory marker, which plays an important role in the formation, progression, and rupture of atherosclerotic plaques and participates in the occurrence and development of cardiovascular diseases. LP-PLA2, also known as platelet-activating factor acetylhydrolase, is a member of the phospholipase family, which is mainly synthesized and secreted by mature macrophages and lymphocytes, and is regulated by other inflammatory mediators. For example, platelet-activating factor can promote its secretion, and interferon and lipopolysaccharide can inhibit its secretion, and interleukin, tumor necrosis factor, and so on, have no obvious effect on its secretion [23, 24]. In the human body, LP-PLA2 mainly exists in the form of binding to lipoprotein particles, and about 2/3 of it is bound to low-density lipoprotein and 1/3 to high-density lipoprotein. It has been reported that LP-PLA2 has antiatherosclerosis function. Platelet-activating factor can promote platelet aggregation in the body, chemotaxis of neutrophils and mononuclear macrophages, and release of inflammatory mediators such as leukotriene, participate in the inflammatory response of the body, and promote the occurrence and progression of atherosclerotic plaques. Platelet-activating factor can be hydrolyzed by LP-PLA2 and then lose its biological activity, reduce the inflammatory response of the body, and have antiatherosclerosis and anti-inflammatory functions [25, 26]. However, most clinical studies show that it mainly participates in the body's inflammatory response and plays a role in promoting the body's inflammatory response. LP-PLA2 can catalyze the hydrolysis of glycerophospholipids on cell membranes and lipoproteins to produce lysophosphatidylcholine and oxidized free fatty acids. The latter two are inflammatory mediators, which can activate inflammatory cells and stimulate the production of adhesion factors and cytokines, thereby inducing monocytes to accumulate under the inner membrane and transform into macrophages. Macrophages swallow oxidized low-density lipoproteins, turn into foam cells, and aggregate to form atherosclerotic plaques, resulting in atherogenic effects. And lysophosphatidylcholine plays a decisive role in the formation and progression of atherosclerosis and participates in the body's inflammatory response, leading to the formation and rupture of plaques, thereby causing secondary cardiovascular events [27, 28].

ST2 is a member of the interleukin-1 receptor superfamily and has immunomodulatory functions. While sST2 is a subtype of ST2, as a decoy receptor, it can be secreted to the outside of the cell and is highly expressed during inflammation and oxidative stress damage. It can affect the increased activation of vascular endothelial growth factor receptor and exposure to vascular endothelial tissue, and it can promote coronary artery disease [29, 30]. sST2 binds to its specific ligand IL-33 to activate the IL-33/ST2L signaling pathway, which is considered to be a mechanical activation system. When myocardial cells are subjected to mechanical stretch stimulation, they will release IL-33 molecules and form receptor complexes with ST2L on the myocardial membrane through paracrine action to activate downstream signaling pathways, thus playing a protective role in the heart by inhibiting inflammatory response and myocardial hypertrophy [31, 32]. sST2, as a competitive receptor of ST2L, can bind to IL-33 released from myocardial tissue cells, then block the cardiac protective effect of the IL-33/ST2L signaling pathway, participate in pathophysiological processes such as inflammatory response and myocardial injury, and regulate the remodeling of the extracellular matrix, leading to a series of cardiovascular negative events [33, 34]. Therefore, when cardiomyocytes are damaged by mechanical stress, such as excessive sST2 in the serum, the myocardial tissue will lack sufficient IL-33 protection, resulting in myocardial remodeling and cardiac dysfunction and promoting the occurrence and development of heart failure. Therefore, it is regarded as a marker of cardiomyocyte hypertrophy and myocardial fibrosis. In recent years, sST2 has become an important research object in the field of heart failure and other cardiovascular diseases, such as coronary heart disease and hypertension, because it is not easily affected by age, body mass index, and kidney function damage.

The results of this study showed that the serum LP-PLA2 and sST2 levels of the observation group were higher than those of the control group, indicating that the serum LP-PLA2 and sST2 levels of AHF patients increased. The reason is that LP-PLA2 is an independent predictor of vascular endothelial injury. Because LP-PLA2 enhances the metabolism of oxidized lipoproteins, the local oxidative pressure increases, which causes damage to vascular endothelial cells and dysfunction and destroys its protective mechanism. The vascular endothelial injury is related to the occurrence and prognosis of AHF. IL-33 is a protein with antimyocardial fibrosis and antiatherosclerosis effects, with which sST2 can antagonize it. sST2 protein is released under the induction of mechanical stress, and the myocardial cells subjected to mechanical stretch can cause the increase of IL-33 and ST2, thus leading to the increase of the serum sST2 level [35, 36]. The results of this study showed that the levels of serum LP-PLA2 and sST2 in the severe group were higher than those in the mild group, and the serum LP-PLA2 and sST2 levels were positively correlated with the disease. These results indicated that the levels of serum LP-PLA2 and sST2 were closely related to the severity of AHF patients and could be used as serum markers to predict the condition of patients. With the aggravation of the disease, the levels of serum LP-PLA2 and sST2 were higher. And the results of this study showed that serum H-FABP and sST2 levels in the event group were higher than those in the no event group. It shows that serum H-FABP and sST2 levels in AHF patients are related to their prognosis.

The ROC curve results in this study showed that the AUC of serum LP-PLA2 and sST2 to predict the prognosis of patients was 0.760 and 0.734, respectively, and the AUC of the two combined to predict the prognosis of patients was 0.811. It shows that the prognostic value of serum LP-PLA2 combined with sST2 is significantly higher than that of single prediction, and it has higher predictive value. Therefore, the detection of serum LP-PLA2 combined with sST2 in patients with AHF can promptly assess the condition and give treatment, which will help improve the prognosis and improve the quality of life of patients.

## 5. Conclusion

Serum LP-PLA2 and sST2 levels were increased in AHF patients, and the levels of LP-PLA2 and sST2 in patients with adverse prognostic events were higher than those without adverse prognostic events. The levels of serum LP-PLA2 and sST2 are closely related to the degree of patients' illness, among which the combined prediction of AHF patients with LP-PLA2 and sST2 has the highest value, which is worthy of promotion.

## Figures and Tables

**Figure 1:** Comparison of serum LP-PLA2 and sST2 levels between the two groups. *Note.* Compared with the control group, ^*∗*^*P* < 0.05.

**Figure 2:** Comparison of serum LP-PLA2 and sST2 levels in patients with different cardiac function grades. *Note.* Compared with the mild group, ^*∗*^*P* < 0.05.

**Figure 3:** Comparison of serum LP-PLA2 and sST2 levels in patients with different prognoses. *Note.* Compared with the event group, ^*∗*^*P* < 0.05.

**Figure 4:** ROC curve of the prognostic value of serum LP-PLA2 and sST2 levels in AHF patients.

**Table 1:** Comparison of general data between the two groups (*n*, $\bar{x}$ ± *s*).

Groups	*n*	Age (years)	Sex	Hypertension	Diabetes	
			Male	Female		
Control group	126	75.96 ± 8.23	92	62	48	20
Observation group	154	76.02 ± 8.48	79	47	72	35
*t/χ* ^*2*^		0.059	0.255	2.121	2.063	
*P*		0.952	0.614	0.145	0.151	

**Table 2:** Correlation between serum LP-PLA2 and sST2 levels and patient's condition.

Predictive indexes	NYHA cardiac function classification	
	*r*	*P*
Serum LP-PLA2 levels	0.804	<0.001
Serum sST2 levels	0.781	<0.001

**Table 3:** The predictive value of serum LP-PLA2 and sST2 levels on the prognosis of patients.

Predictive indexes	AUC	95% CI	Youden index	Sensitivity (%)	Specificity (%)	Cutoff value
LP-PLA2	0.760	0.680–0.840	0.402	95.3	44.9	165.42 ng/ml
sST2	0.734	0.649–0.818	0.379	76.7	61.2	82.62 pg/ml
Combined prediction	0.811	0.738–0.884	0.513	86.0	65.3	—

## Data Availability

The data used to support the findings of this study can be obtained from the corresponding author upon reasonable request.
